This article has been retracted.

# Correlation of *CCNA1* Promoter Methylation with Malignant Tumors: A Meta-Analysis Introduction

**DOI:** 10.1155/2015/134027

**Published:** 2015-01-15

**Authors:** Bin Yang, Shuai Miao, Le-Ning Zhang, Hong-Bin Sun, Zhe-Nan Xu, Chun-Shan Han

**Affiliations:** ^1^Department of Thoracic Surgery, China-Japan Union Hospital of Jilin University, Changchun 130033, China; ^2^Department of Geriatrics, China-Japan Union Hospital of Jilin University, Changchun 130033, China

## Abstract

Epigenetic silencing of tumor suppressor genes by promoter methylation plays vital roles in the process of carcinogenesis. The purpose of this meta-analysis was to determine whether the aberrant methylation of cyclin A1 (*CCNA1*) may be of great significance to human malignant tumors. By searching both English and Chinese language-based electronic databases carefully, we tabulated and analyzed parameters from each study. All human-associated case-control studies were included providing available data for *CCNA1* methylation and reporting the adjusted odds ratios (ORs) and 95% confidence intervals (CI) conducted with the use of Version 12.0 STATA software. A total of 10 case-control studies (619 patients with cancers and 292 healthy controls) were included for the following statistical analysis. Pooled OR values from all articles revealed that the frequency of *CCNA1* methylation in cancer tissues was significantly higher than those of normal tissues (*P* < 0.001). Further ethnicity indicated that the frequency of *CCNA1* methylation was correlated with the development of malignant tumors among all those included experimental subgroups (all *P* < 0.05). These data from results indicated a significant connection of *CCNA1* methylation with poor progression in human malignant tumors among both Caucasian and Asian populations.

## 1. Introduction

Cancer, as the leading cause of mortality in developed countries, refers to a variety of malignant diseases containing abnormal cell growth with the possibility to invade or migrate to other parts of the body, with lung, prostate, colorectal, and stomach cancers being prevalent in males and breast, colorectal, lung, and cervical cancers being common in females [1]. Clinically, cancer is possibly characterized by a new lump, abnormal bleeding, a prolonged cough, unexplained weight loss, and a change in bowel movements [2]. It has been reported that approximately 14.1 million new cancer cases were diagnosed worldwide in 2012, responsible for 8.2 million deaths, equivalent to 14.6% of all human deaths (World Cancer Report Fund/American Institute for Cancer Research: Food, Nutrition, Physical Activity, and the Prevention of Cancer: a Global Perspective, Washington, DC: AICR, 2007). In addition, about 1,660,290 new cases of cancer and 580,350 cancer deaths are estimated to have occurred in the US in 2013 [3]. It is widely accepted that the pathogenesis of cancers is regarded to be complicated involving both genetic and environmental influences [4, 5]. Various risk factors may be implicated in cancer etiology, including obesity, lack of physical activity, drinking, smoking, a poor diet, and exposure to ionizing radiation [4, 6–8]. Recent evidence has demonstrated that methylation of* cyclin A1 (CCNA1)* gene may also considerably conduce to the process of tumorigenesis [9, 10].

*CCNA1* belongs to the highly conserved cyclin family, which are manifested by a dramatic periodicity in protein abundance via the cell division cycle and function as activating subunits of enzymatic complex in combination with cyclin-dependent kinases (CDKs) [11].* CCNA1* is capable of targeting activated cell division cycle 2 and cyclin-dependent kinase 2 to substrates essential for condensation of chromatin and other alterations in morphology during the process of apoptosis [12]. In general, the expression of* CCNA1* is tissue-specific and high* CCNA1* expression is limited to testis; besides, lower levels of* CCNA1* expression are also observed in other human cell lines and in healthy brain [13]. Currently,* CCNA1* expression has been illustrated to be downregulated in various tumors, including head and neck squamous-cell cancer (HNSCC) and nasopharyngeal carcinoma; and the promoter of the* CCNA1* gene is found to be frequently methylated in colon cancer and HNSCC [14–16]. Human* CCNA1* gene has been mapped to chromosome 13q12.3-q13, consisting of 9 exons and 8 introns and extending over approximately 13 kb in length [17, 18]. It has been widely described in several studies that* CCNA1* may be an important tumor suppressor gene and plays a crucial part in head and neck carcinoma and cervical and nasopharyngeal cancers [12, 19, 20]. More importantly, promoter methylation of tumor suppressor genes including* CCNA1* gene may conduce to an immortalized phenotype via silencing expression of genes which possess the ability to control cell differentiation or suppress cell growth [9]. From this aspect, we postulated that* CCNA1* gene promoter methylation may lead to tumor cell proliferation in the development of cancers. In a precious study, promoter methylation of* CCNA1* gene is found in 45% of tumors but in none of the normal tissues, suggesting the implication of* CCNA1* gene methylation in carcinogenesis [12]. Furthermore, a relatively high frequency of methylation* CCNA1* gene was observed in bladder cancer tissues but not in normal uroepithelium, revealing that* CCNA1* gene promoter methylation may participate in the pathogenesis of bladder cancer [5]. Nevertheless, there still existed discordant findings with regard to the role of* CCNA1* gene methylation in tumorigenesis [21, 22]. Hence, the present meta-analysis was carried out to explore the plausible impact of* CCNA1* gene methylation on cancer development.

## 2. Materials and Methods

### 2.1. Data Sources and Keywords

To identify all pertinent papers that assessed the correlations of* CCNA1* methylation with malignant tumors, we comprehensively searched PubMed, Embase, Web of Science, Cochrane Library, CISCOM, CINAHL, Google Scholar, CBM, and CNKI databases (last updated search on May 1, 2014), utilizing selected common keywords regarding the* CCNA1* protein and tumor. As for the keywords to be applied in our initial literature search, we selected (“*CCNA1* protein, human” or “*CCNA1*” or “cyclin A1” or “cyclin A1 protein” or “Cyclin-A1”) and (“Methylation” or “DNA Methylation” or “Hypermethylation” or “demethylation”) for the exposure factors. In addition, (“Neoplasms” or “Neoplasm” or “Cancer” or “Cancers” or “carcinomas” or “carcinoma” or “tumor” or “tumors”) were selected as the outcome factors. No restriction was set to the language of the article. We also further scanned the bibliographies of relevant articles manually to identify additional potential relevant papers. When the enrolled papers supplied unclear additional data in their original publications, the first authors would be contacted and asked for clarifications.

### 2.2. Selection Criteria

We searched throughout for all human-associated case-control studies providing available data for* CCNA1* methylation, including patients with malignant tumors and normal controls, and reporting the adjusted odds ratios (ORs) and 95% confidence intervals (CI). We just extracted studies supplying the sample number and sufficient information about* CCNA1* methylation and excluded those articles with incomplete unavailable or inappropriate clinicopathologic data or those regarding tumors not confirmed by histopathologic examinations. In addition, only the studies with the minimum number of samples greater than 30 were enrolled. However, when the extracted studies had subjects overlapping more than 50% with two or more papers, we merely enrolled the one whose population was the most comprehensive. At the same time, only the newest or complete study was included when the extracted studies were published by the same authors or groups, after careful reexamination.

### 2.3. Data Extraction

In order to reduce the bias and enhance the credibility, two investigators extracted information from the retrieved papers according to the selection criteria separately and arrived at a consensus on all the items through discussion and reexamination. The following relevant data were extracted from eligible studies prospectively in the final analyses: surname of first author, year of publication, source of publication, study type, study design, source of samples, sample size, age, sex, ethnicity and country of origin, disease type, detection method for* CCNA1* methylation, and methylation of* CCNA1* in cancer tissues and normal tissues. All authors approved the final determinant of the studies to be enrolled.

### 2.4. Quality Assessment

To decide whether the study in question is of high quality, the two authors used a set of predefined criteria based on the REMARK guidelines and Newcastle-Ottawa Scale (NOS) criteria to assess the studies independently [23, 24]. The REMARK guidelines, consisting of 20 detailed items, assess several aspects of the enrolled studies, such as study aim, study design, patient enrollment, biomarker detection, statistical analysis method, and report of results. On the other hand, the NOS criteria are scored based on three aspects: (1) subject selection: 0~4; (2) comparability of subject: 0~2; (3) clinical outcome: 0~3. Total NOS scores range from 0 (lowest) to 9 (highest). According to the NOS scores, the included studies were classified into two levels: low quality (0–6) and high quality (7–9), respectively. Discrepancies on NOS scores of the enrolled articles were resolved by discussion and consultation with the third reviewer.

### 2.5. Statistical Analysis

To calculate the effect size for each study, the summary ORs with 95% CI were used for cancer tissue versus normal tissue categories of* CCNA1* methylation with the utilization of *Z* test. In order to supply quantitative evidence of all selected studies and minimize the variance of the summary ORs with 95% CI, we conducted the current statistical meta-analyses by utilizing a random-effects model (DerSimonian and Laird method) or a fixed-effects model (Mantel-Haenszel method) of individual study results under the situation where data from independent studies could be combined. Random-effects model was applied when heterogeneity existed among studies, while fixed-effects model was applied when there was no statistical heterogeneity. The subgroup meta-analyses were also conducted by ethnicity, disease type, sample size, and detection method to explore potential effect modification, and heterogeneity across the enrolled studies was evaluated by Cochran's *Q*-statistic (*P* < 0.05 was regarded as statistically significant) [25]. As a result of low statistical power of Cochran's *Q*-statistic, *I* ^2^ test was also measured to reflect the possibility of heterogeneity between studies [26]. The *I* ^2^ test values ranged from 0% (no heterogeneity) to 100% (maximal heterogeneity). The one-way sensitivity analysis was performed to evaluate whether the results could have been affected significantly through deleting a single study in our meta-analysis one by one to reflect the influence of the individual data set on the pooled ORs. The funnel plot was constructed to assess publication bias which might affect the validity of the estimates. The symmetry of the funnel plot was further evaluated by Egger's linear regression test [27]. All tests were two-sided and a *P* value of <0.05 was regarded as statistically significant. To make sure that the results are credible and accurate, two investigators inputted all information in the STATA software, Version 12.0 (StataCorp, College Station, TX, USA), separately and arrived at an agreement.

## 3. Results

### 3.1. Included Studies

Our present meta-analysis hit a total of 10 case-control studies that provided information on the correlation of* CCNA1* methylation with tumors [5, 9, 10, 12, 19–22, 28, 29]. Seven studies were conducted in populations of Asian descent and 4 in populations of Caucasian descent, including 911 subjects in total (619 patients with cancers and 292 healthy controls), which were published between 2003 and 2014. The characteristics and methodological quality of the extracted studies were presented in Table 1. The countries where the studies were performed were Brazil, China, Germany, The Netherlands, Thailand, USA, and Korea. The sources of samples in our present meta-analysis were all from tissues. Diseases involved in our meta-analysis consist of head and neck squamous-cell carcinoma (HNSCC), colorectal cancer (CC), nasopharyngeal carcinoma (NPC), bladder cancer (BCa), and hepatocellular carcinoma (HCC). The methods detecting* CCNA1* methylation in this current meta-analysis included MSP (*n* = 5), qMSP (*n* = 3), and Duplex MSP (*n* = 2). Additionally, as for the step of screening, a flow chart of the study selection process was displayed in Figure 1. Initially, a total of 80 papers were selected from the 9 databases through screening the title and keywords. After excluding the duplicates (*n* = 2), letters, reviews, or meta-analyses (*n* = 9), nonhuman studies (*n* = 13), and the studies not related to research topics (*n* = 20), the remaining studies (*n* = 36) were reviewed and additional 23 studies were excluded for not being case-control or cohort study (*n* = 4), relevant to* CCNA1* (*n* = 7), or relevant to cancer (*n* = 12). After the remaining 13 trials were further reviewed, 10 papers were enrolled in the final analysis. During the final selection process, the major reason for abandon was not supplying enough information (*n* = 3). All quality scores of the included studies were higher than 6 (high quality). From 2001 to 2014, the number of articles selected from those electronic databases was shown in Figure 2.

### 3.2. Association of* CCNA1* Methylation with Cancers

As shown in Figure 3, the major findings of the present meta-analysis revealed a higher* CCNA1* methylation level in patients with cancers compared to that in normal controls (OR = 12.45, 95% CI: 6.35–24.42, and *P* < 0.001). Subgroup analysis based on ethnicity implied that* CCNA1* methylation level was higher in cancer tissues than in normal tissues in both Caucasians and Asians (all *P* < 0.05) (Figure 4). In addition, subgroup analysis by disease type implicated that methylation level of* CCNA1* in cancer tissues was higher than that in normal tissues in all HNSCC, CC, NPC, BCa, and HCC subgroups (all *P* < 0.05). Subgroup analysis based on sample size revealed that the* CCNA1* hypermethylation occurred more frequently in the cancer tissues relative to the normal tissues; in the large sample size subgroup, similar association was also observed in the small sample size subgroup (all *P* < 0.05). Further subgroup analysis based on detection method implied that* CCNA1* methylation level in patients with cancers was higher than that in the normal controls by using qMSP, MSP, and Duplex MSP (all *P* < 0.05).

### 3.3. Sensitivity Analysis and Publication Bias

A leave-one-out sensitivity analysis was carried out to evaluate whether a particular study or studies would lead to heterogeneity and impact on the pooled ORs for* CCNA1* methylation level. The overall statistical significance does not change when any single study was omitted. Therefore, the current meta-analysis data is relatively stable and credible (Figure 5). The graphical funnel plots of those 11 studies appear to be symmetrical, and Egger's test showed no publication bias (both *P* > 0.05) (Figure 6).

## 4. Discussion

Our meta-analysis was conducted to clarify the relationship of* CCNA1* methylation and the development of tumors. The main results in the current study showed a higher* CCNA1* methylation level in cancer patients than that in normal controls, indicating that the methylation of* CCNA1* may have a significant connection with the development of human tumors, including HNSCC, NSCLC, CC, NPC, BCa, and HCC. CCNA1, also called cyclin A1, could bind to many cell cycle regulators like transcription factor E2F-1, Rb, and p21 family proteins to regulate the cell apoptosis, accompanied with CDK kinases to arrest G2M phases and interact with Ku70 to repair the DNA double-strand break [12, 30–32]. The abnormal methylation of* CCNA1* gene, especially in the CpG islands of gene promoter, could block the transcription, thus affecting the expression of CCNA1, which may lead to CCNA1 dysfunctions in cell differentiation and cell growth, contributing to the progression of many human tumors, such as HNSCC, NSCLC, CC, NPC, BCa, and HCC [9, 10, 20, 33–35]. The hypermethylation of promoter in the* CCNA1* gene was found in the saliva and plasma of patients suffering from HNSCC, while the frequency of* CCNA1* hypermethylation decreased significantly after treatment, indicating that* CCNA1* gene hypermethylation may be an essential reason for HNSCC development [29].* CCNA1* gene hypermethylation might hinder its antitumor function in regulating the cell apoptosis by binding cell cycle regulators like transcription factor E2F-1, Rb, and p21 family proteins as we mentioned before, which is thus related to the development of NSCLC, NPC, BCa, and HCC (http://www.i-md.com/docsearch/doc/edbe90ca-14a0-4780-8286-7fa6e0be1b51?dp=Respiratory) [5, 20, 21]. In addition, as a potential suppressor gene for epithelial tumors,* CCNA1* could participate in the TP53 activation in the CC patients by viral protein and host protein interaction;* CCNA1* gene hypermethylation of promoter is more frequently found in invasive CC compared to that in squamous-cell CC, suggesting its role as an effective marker for invasive CC diagnosis [19]. To confirm our analysis, we found similar conclusion from the study of Rettori et al. They showed that* CCNA1* was frequently hypermethylated in HNSCC patients with second primary tumors and thus could be used as a potent marker for neoplastic evolution [36]. To evaluate the influence of ethnicity, different kinds of diseases, sample size, and methylation detection method on the relationship between* CCNA1* methylation and tumors development, a further deep stratified analysis was performed. We could observe no obvious effect of ethnicity and methylation detection method on the relationship, which demonstrated the subjectivity and reasonability of our analysis.

A number of potential limitations have been taken into account in our meta-analysis. First and foremost, it was widely acknowledged that methylation analysis depended mostly on harvested cells; in this regard, it was easier to ignore the issue of sampling error. Besides, there was a lack of an accepted gold standard against which to compare methylation results, thereby having a strong influence on the reliability of the further investigation in this field. Secondly, although there was no heterogeneity existing in ethnicity, different kinds of diseases, sample size, and methylation detection methods in our subgroup analysis, other different types of heterogeneity sources should be better to be presented among all the included studies. A third limitation of this analysis may be the publication and reporting bias which may be existent. We attempted to use several Chinese and English databases as complete as possible for the purpose of minimizing publication bias; however, we did not take unpublished papers and abstracts into account entirely. Fourthly, in some of the included literatures, the number of cancer patients or healthy controls was relatively small, which may restrict the outcome of this meta-analysis. Finally, it is difficult to determine the cut-off point of* CCNA1* hypermethylation for predicting cancer risk, and thereby the sensitivity and specificity of genes methylation respecting cancer risks could not be easily decided.

To sum up, the findings of our meta-analysis demonstrated that* CCNA1* was frequently and specifically hypermethylated in several cancer samples, suggesting that the aberrant methylation of* CCNA1* was significantly related to the development of human cancers, especially visible in HNSCCCC and NPC in the general populations. However, it is essential to carry out a more extensive larger scale study with larger patient groups and longer follow-up period for further validation.

## Figures and Tables

**Figure 1:** Flow chart shows study selection procedure. Eleven case-control studies were included in this meta-analysis.

**Figure 2:** Distribution of the number of topic-related literatures in electronic databases over the last decade.

**Figure 3:** Forest plot for the associations between aberrant* cyclin A1* promoter methylation and the pathogenesis of human tumors.

**Figure 4:** Subgroup analyses of the relationships between aberrant* cyclin A1* promoter methylation and the pathogenesis of human tumors.

**Figure 5:** Sensitivity analysis of the summary odds ratio coefficients on the associations between aberrant* cyclin A1* promoter methylation and the pathogenesis of human tumors.

**Figure 6:** Funnel plot of publication biases on the associations between aberrant* cyclin A1* promoter methylation and the pathogenesis of human tumors.

**Table 1:** Characteristics of included studies focused on methylation ratio of* CCNA1. *

First author	Year	Ethnicity	Disease	Sample	Number			Gender (M/F)	Age (years)	Method	NOS score
					Tumor	Benign	Normal				
Longo [29]	2014	Caucasians	HNSCC	Tissue	96	0	79	75/21	59 (20~90)	qMSP	8
Liu [28]	2013	Asians	CC	Tissue	40	0	40	0/40	—	MSP	6
Weiss [10]	2011	Caucasians	HNSCC	Tissue	49	0	31	—	63.7 ± 11.8	MSP	7
Yang [9]	2010	Caucasians	CC	Tissue	60	40	20	—	46 (38~57)	qMSP	7
Yanatatsaneejit [20]	2008	Asians	NPC	Tissue	46	0	20	—	—	Duplex MSP	6
Brait [5]	2008	Caucasians	BCa	Tissue	93	0	26	—	67 (39~83)	qMSP	8
					25	0	5	—	66 (34~84)	qMSP	
Yu [21]	2003	Asians	BCa	Tissue	132	23	0	107/25	—	MSP	8
Kitkumthorn [19]	2006	Asians	CC	Tissue	30	24	25	—	—	Duplex MSP	6
Tokumaru [12]	2004	Asians	HNSCC	Tissue	20	0	11	—	—	MSP	6
Yu [21]	2003	Asians	HCC	Tissue	28	0	28	—	—	MSP	6

M: male; F: female; NOS: Newcastle-Ottawa Scale; HNSCC: head and neck cancer; NSCLC: non-small-cell lung cancer; CC: choriocarcinoma; NPC: nasopharyngeal carcinoma; BCa: bladder cancer; HCC: hepatocellular carcinoma; MSP: methylation specific PCR.
